# Use of Traditional Chinese Medicine and Its Impact on Medical Cost among Urban Ischemic Stroke Inpatients in China: A National Cross-Sectional Study

**DOI:** 10.1155/2021/8554829

**Published:** 2021-10-29

**Authors:** Zhengwei Huang, Xuefeng Shi, Stephen Nicholas, Elizabeth Maitland, Yong Yang, Weihan Zhao, Yong Ma, Yan Jiang

**Affiliations:** ^1^School of Management, Beijing University of Chinese Medicine, Beijing, China; ^2^National Institute of Traditional Chinese Medicine Strategy and Development, Beijing University of Chinese Medicine, Beijing, China; ^3^Australian National Institute of Management and Commerce, Eveleigh Sydney, NSW 2015, Australia; ^4^School of Economics and School of Management, Tianjin Normal University, Tianjin, China; ^5^Guangdong Institute for International Strategies, Guangdong University of Foreign Studies, Guangzhou, China; ^6^Newcastle Business School, University of Newcastle, Newcastle, Callaghan, Australia; ^7^School of Management, University of Liverpool, Chatham Building, Chatham Street, Liverpool L697ZH, UK; ^8^Medical Device Regulatory Research and Evaluation Center, West China Hospital, Sichuan University, Chengdu, China; ^9^China Health Insurance Research Association, Beijing, China

## Abstract

**Background:**

Traditional Chinese medicine (TCM) has long been widely adopted by the Chinese people and has been covered by China's basic medical insurance schemes to treat ischemic stroke. Previous research has mainly highlighted the therapy effect of TCM on ischemic stroke patients. Some studies have demonstrated that employing TCM can reduce the medical burden on other diseases. But no research has explored whether using TCM could reduce inpatient medical cost for ischemic stroke in mainland China. The purpose of this study is to investigate the impact of the use of TCM on the total inpatient cost of ischemic stroke and to explore whether TCM has played the role of being complementary to, or an alternative for, conventional medicine to treat ischemic stroke.

**Methods:**

We conducted a national cross-sectional analysis based on a 5% random sample from claims data of China Urban Employee Basic Medical Insurance (UEBMI) and Urban Resident Basic Medical Insurance (URBMI) schemes in 2015. Mann–Whitney test was used to compare unadjusted total inpatient cost, conventional medication cost, and nonpharmacy cost estimates. Ordinary least square regression analysis was performed to compare demographics-adjusted total inpatient cost and to examine the association between TCM cost and conventional medication cost.

**Results:**

A total of 47321 urban inpatients diagnosed with ischemic stroke were identified in our study, with 92.6% (43843) of the patients using TCM in their inpatient treatment. Total inpatient cost for TCM users was significantly higher than TCM nonusers (USD 1217 versus USD 1036, *P* < 0.001). Conventional medication cost was significantly lower for TCM users (USD 335 versus USD 436, *P* < 0.001). The average cost of TCM per patient among TCM users was USD 289. Among TCM users, conventional medication costs were found to be positively associated with TCM cost after adjusting for confounding factors (Coef. = 0.144, *P* < 0.001).

**Conclusion:**

Although the use of TCM reduced the cost of conventional medicine compared with TCM nonusers, TCM imposed an extra financial component on the total inpatient cost on TCM users. Our study suggests that TCM mainly played a complementary role to conventional medicine in ischemic stroke treatment in mainland China.

## 1. Background

Stroke is one of the world's most serious chronic diseases due to the severity of its health damage and to its catastrophic health costs. In 2017, there were approximately 104 million stroke patients, with an estimated 13 million new global cases in 2020. Stroke claimed over 6 million lives in 2017, becoming the third leading cause of both death and disability-adjusted life-years (DALYs) [1, 2]. The health care expenditure spent on stroke imposed a significant economic burden on health systems, estimated at over €27 billion in Europe alone in 2020 [3], and imposed a heavy financial burden on families with stroke victims, especially in low- and middle-income countries [1].

Stroke has been the leading cause of both death and DALYs in China, with an estimated 1.1 million stroke-related deaths in 2013 or about 15% of the global total of 6 million stroke deaths [4, 5]. Among various types of stroke, ischemic was the main subtype in China [6]. A recent study revealed that the weighted average 2013–2016 annual total medical cost of stroke was RMB10637 (USD1707.82), with inpatient costs accounting for 94% (RMB10034 or USD1586) of total stoke medical costs, with medication costs accounting for 50.6% of average stroke-related medical costs [6]. While Chinese stroke patients mainly receive conventional modern medicine in their treatment, it has been claimed that conventional medicine fails to some degree to optimally treat or reduce costs of stroke [7–9].

Traditional, complementary, and alternative medicine (TCAM) is regarded as both a complement and an alternative to conventional stroke treatment for its equitability, accessibility, and low cost. Previous studies show that 46% of stroke patients in the United States [10], 66% in Malaysia [11], 36% in Indian [12], and 54% in Korea [13] have used TCAM stroke treatments. Evidence suggests that more than half of stroke patients who received TCAM treatment benefited, including improved stroke symptoms, walking patterns, psychological distress, limb strength, and standing balance [12, 14]. Traditional Chinese medicine (TCM), one specific type of TCAM, has been used for the treatment of stroke in China for thousands of years, due to its safety, lower cost, effectiveness, and convenience [15]. The *Healthy China 2030 Program* has stressed the uniqueness and importance of TCM in prevention, rehabilitation, and treatment for severe diseases, including stroke. Studies have shown that TCM stroke treatment can promote angiogenesis, strengthen neurological function, improve stroke recovery, advance life quality, and lower recurrence risk through its nonmedication therapies, herbal medicines, and pharmaceutical preparations [5, 16–25]. Using a Taiwanese National Health Insurance (NHI) database, Su et al. [26] found that, among patients with uterine fibroid, TCM use correlated negatively with consumption of conventional medicine and decreased total medical costs. Tsai et al. [27] also demonstrated that, among patients with heart failure, the hospital cost was lower for TCM users than for TCM nonusers. Both studies suggested that TCM could be a substitute for conventional medicine to treat diseases and with lower healthcare costs.

Given the partial evidence of lower cost and effectiveness of TCM ischemic stroke treatment, do TCM stroke treatment users consume fewer conventional medications and incur lower medical cost than conventional-only stroke treatment users? Unfortunately, few studies have investigated the impact of the use of TCM on medical cost in mainland China. This study investigates the impact of the use of TCM on total inpatient medical costs of ischemic stroke sufferers and explores whether TCM was a complement or an alternative for conventional ischemic stroke treatments from a cost perspective.

## 2. Materials and Methods

### 2.1. Data Source

Our data come from a 5% random sample of the Urban Employee Basic Medical Insurance (UEBMI) and the Urban Resident Basic Medical Insurance (URBMI) beneficiaries' insurance claims, which used a stratified random sample design and were conducted in 2015 by China Health Insurance Research Association (CHIRA) [28]. UEBMI and URBMI were the two main social health insurance schemes administered by China government, covering more than 95% of the urban residents, for roughly 750 million, or 53%, of the total Chinese population in 2015 [29, 30]. Based on contributions from employers and employees, UEBMI, launched in 1998, offers compulsory and comprehensive insurance for employed people with a per capita fund of RMB3144 (USD505) in 2015, with an 80% reimbursement rate and basic urban wage reimbursement ceiling. Based on a government subsidy and individual premiums, URBMI, started in 2007, is voluntary, offering limited insurance to the unemployed, retired, students, and children among urban residents, with a per capita fund of RMB560 (USD 90) in 2015, with a 70% reimbursement rate and farmer income-based reimbursement ceiling [31]. These cross-sectional data consist of ischemic stroke patients' demographic information (sex and age), diagnosis (classified according to International Classification of Diseases, 10th edition (ICD-10)), length of hospital stay (LOS), hospital level (primary, secondary, and tertiary), hospital type (TCM and non-TCM), economic region (east, west, and central), type of medical insurance expenditure (URBMI and UEBMI), and inpatient cost of hospital treatment.

### 2.2. Samples

According to the International Classification of Diseases, 10th version (ICD-10) codes, all patients whose primary diagnosis was ischemic stroke (ICD-10: I63.X) between January 2015 and December 2015 were included. Inclusion criteria for the inpatients with ischemic stroke were at least one inpatient claim with a primary diagnosis of ICD-10: I63.X code (defined as the “ischemic condition of the brain, producing a persistent focal neurological deficit in the area of distribution of the cerebral arteries” [32]) in 2015. Patients were excluded when their data were incomplete or logically erroneous when calculating medical costs, such as when individual total medical costs were not equal to the sum of medication cost and nonpharmacy cost. We identified 47321 ischemic stroke patients in the 2015 CHIRA claims database.

### 2.3. Measures

According to the CHIRA claims data, TCM treatment included three subtypes, Chinese herbal medicine (H), Chinese patent medicine (P), and Chinese medicine injection (J). TCM users were defined by inpatients who utilized any kind of the three TCM treatments. TCM users frequently received conventional medicines as well as TCM treatments. TCM nonusers were defined as patients who did not receive any type of TCM treatment. We also extracted information on 8 prevalent comorbidities among ischemic stroke patients [33], comprising hypertension, coronary heart disease, diabetes, chronic pulmonary disease, peripheral vascular disease, other neurological diseases, rheumatoid arthritis, and peptic ulcer disease.

Medical inpatient costs comprised conventional medication pharmacy costs, TCM medication pharmacy costs, and nonpharmacy costs. Except for the costs of TCM and conventional prescription drugs, the nonpharmacy cost referred to all other inpatient costs, including diagnostic tests and nonmedication therapy. The inpatient cost was calculated for each patient for the whole year of 2015. When a patient was admitted more than once during 2015, costs for each admission were summed to obtain the inpatient cost. All patients leaving hospital from January 1, 2015, to December 31, 2015, were considered as the index event. Given the data source, an individual's 2014 hospital costs before the index event were included in an individual's 2015 hospital costs. All costs were based on a constant 2015 US$1.0 = RMB 6.2284 annual average exchange rate.

### 2.4. Statistical Analysis

Descriptive statistics (percentage and median with interquartile range (IQR)) were used to describe the demographic information and hospital costs. Demographic variables and comorbidities between TCM users and TCM nonusers were examined using chi-square tests. Since the value of medical expenditures usually has a skewed distribution, the Mann–Whitney test was used to identify the differences in inpatient costs between TCM users and TCM nonusers. To quantify the difference in total inpatient cost between TCM users and TCM nonusers, an ordinary least squares regression analysis was conducted, in which the dependent variable was the logarithm of total inpatient cost and the independent variable was the use/nonuse of TCM for each patient, adjusted for the confounding variables, including length of hospital stay (LOS), sex, age, type of medical insurance, hospital level, type of hospital, region, and comorbidities, which can influence both the dependent and independent variable. A further ordinary least squares regression analysis was performed to investigate the association between TCM cost and conventional medication cost, with the logarithm of TCM cost as the dependent variable and logarithm of conventional medication cost as the independent variable of interest, adjusted for the confounding factors described above. A two-sided *P* value less than 0.05 was considered statistically significant. All analyses were performed using STATA/SE 15.

## 3. Results

### 3.1. Basic Characteristics

As shown in Table 1, 47321 patients suffered ischemic stroke, where 7.4% (3478) did not use any TCM treatment (TCM nonusers) and 92.6% (43843) used at least one type of TCM treatment (TCM users), comprising Chinese herbal medicine, Chinese patent medicine, and Chinese medicine injection. Table 1 shows that 56.6% (26795) of ischemic stroke inpatients were male, but the proportion of female TCM users (43.7%) was significantly higher than TCM nonusers (39.7%) (*P* < 0.001). The median age of our sample was 68 years; 63.3% (29950) of patients participated in the UEBMI scheme; 14.8% of patients received medical treatment in TCM hospitals, but significantly more TCM users were treated in TCM hospitals (15.1%) than TCM nonusers (11.2%) (*P* < 0.001). From Table 1, 31.7% of TCM users were treated in tertiary hospitals and 19.6% in primary hospitals, while 39.7% of TCM nonusers were treated in tertiary and only 14.4% in primary hospitals (*P* < 0.001). TCM users were mainly from the central region (46.7%), followed by the eastern region (34.7%), but TCM nonusers were roughly equally treated in the central (42.8%) and eastern (40.5%) regions (*P* < 0.001). The proportions of patients who had comorbidities, such as hypertension, coronary heart disease, diabetes, chronic pulmonary disease, peripheral vascular disease, other neurological diseases, rheumatoid arthritis, and peptic ulcer disease, were all significantly higher among TCM users than TCM nonusers (*P* < 0.001). Finally, the average length of stay (ALOS) for TCM users (15.1 days) was significantly lower than TCM nonusers (17.7 days) (*P* < 0.001).

### 3.2. Inpatient Cost between TCM Users and TCM Nonusers Associated with Demographic Characteristics

Table 2 reveals the differences in TCM user and TCM nonuser ischemic stroke inpatient medical costs. Overall, the median total inpatient cost for TCM users was RMB7579 (USD1217), significantly higher than TCM nonusers (RMB6455 (USD1036)) (*P* < 0.001). TCM users' significantly higher inpatient cost than TCM nonusers differed according to sex, insurance type, TCM hospital, and region (all *P* < 0.001). Inpatient cost of TCM users over 30 years old and TCM users admitted to secondary hospitals and tertiary hospitals had significantly higher medical costs than TCM nonusers. In addition, TCM users with comorbidities of hypertension, coronary heart disease, diabetes, and other neurological diseases had significantly higher inpatient cost than TCM nonusers.

### 3.3. Analysis of Inpatient TCM Users and TCM Nonusers Medical Costs

To further examine the difference in inpatient medical cost between TCM users and TCM nonusers, we conducted a multivariate regression analysis after the confounding variables were fixed.  Table 3 reveals that TCM users incurred a 32.5% (Coef. = 0.325, *P* < 0.001) higher medical cost compared to TCM nonusers after adjusting for length of stay (LOS), age, sex, insurance type, hospital type, region, and comorbidities.

### 3.4. Composition of TCM Users and TCM Nonusers Inpatient Medical Costs

Table 4 compares the composition of inpatient cost of TCM nonusers and TCM users, which helps explain the reason why TCM users faced a higher inpatient medical cost component. As categorized in the insurance payment system, inpatient medical cost for ischemic stroke inpatients were divided into conventional medication costs, TCM medication costs, and nonpharmacy medical costs. From the payment data in Table 4, there was no significant difference in nonpharmacy medical cost between TCM users and TCM nonusers (*P* > 0.290). While ischemic stroke TCM users incurred RMB629/USD101 lower conventional medication cost (RMB2087/USD335) compared to TCM nonusers (RMB2716/USD436) (*P* < 0.001), TCM medication costs (RMB1803/USD289) meant that total medication costs of TCM users (RMB4175/USD670) were higher than TCM nonusers medication costs (RMB2716/USD436) (*P* < 0.001).

### 3.5. Multivariate Regression Analysis to Examine the Association of TCM Cost

Table 4 shows that the use of TCM imposed a substantial medical cost component on TCM users. A multiple regression analysis in Table 5 modeled the association between TCM costs and conventional medication costs for TCM users, which showed a positive association of TCM costs with conventional medication costs (Coef. = 0.144, *P* < 0.001). Among TCM users, TCM medication cost significantly increased with the prescription of conventional medicine, demonstrating that TCM treatments were complements, rather than substitutes, to conventional treatment.

## 4. Discussion

Traditional Chinese medicine (TCM) was a treatment sought out by ischemic stroke patients and made available by healthcare providers. To our knowledge, this is the first study using a large nationwide Chinese health insurance claims database to explore whether using TCM could reduce medical cost for ischemic stroke inpatients. Compared with patients who did not use any kind of TCM (7.4%), the majority of ischemic stroke patients utilized some TCM treatments (92.6%), which was much higher than TCM use in other countries that used TCM in the stroke treatment [10–13]. Also, complementary and alternative medications were less expensive than conventional medications [26, 34, 35]. While TCM users incurred lower conventional medication costs than TCM nonusers, we found that inpatient TCM users' medical costs were 32.5% higher than those of TCM nonusers after adjusting for LOS, age, sex, insurance type, hospital type, region, and comorbidities.

While total inpatient medical cost was significantly higher for TCM users, we found that the use of TCM reduced on average the cost of conventional medication use by RMB629/USD101 compared with TCM nonusers. This small TCM impact on conventional medication costs suggests that TCM attenuates to some extent conventional medication costs. However, the average costs of TCM medication (RMB1803/USD289), plus the use of conventional medications (RMB2087/USD335), meant that the total cost of medication for TCM user ischemic stroke inpatients was significantly higher (RMB4175/USD670) than TCM nonusers who only used conventional medication (RMB2716/USD436). As a result, the extra medication cost of TCM users imposed a significant financial composition, roughly an additional 32.5%, compared to the total medical cost of TCM nonusers. These data suggest that TCM was complementary, rather than a substitute, for conventional medical treatment for ischemic stroke inpatients.

Previous studies showed that TCM mainly played a role in the recovery period of ischemic stroke treatment. Although randomized clinical trials and animal studies have confirmed that TCM, specifically Chinese patent medicine, Chinese herbal medicine, and Chinese medicine injection, is effective in treating ischemic stroke [36–39], conventional recombinant tissue plasminogen activator is almost the only approved and available thrombolytic agent used at the onset of acute ischemic stroke [40, 41]. As reported by both clinical trials [25, 40] and real-world studies [42, 43], the effectiveness and safety of TCM were mostly related to the ischemic stroke rehabilitation and recovery of motor function stages. There is no TCM medication to replace conventional thrombolytic medication during the onset of acute ischemic stroke.

TCM cost was positively associated with conventional medication cost after adjusting for the confounding factors. The use of TCM and conventional medicine altogether increased total inpatient cost among TCM users, revealing that TCM was complementary rather than an alternative for conventional medicine during the whole stroke treatment. This might be explained from both the demand and supply sides. From the demand side, patients in Asian countries, especially China, have a strong cultural belief in TCM, seeking additional TCM medication therapy and demanding TCM prescriptions [44, 45]. From the supply side, the drug markup policy and bonus system, which rewarded physicians based on the monetary values of drugs they prescribed, encouraged physicians to overprescribe drugs [46]. The zero-markup policy for conventional drugs, which was introduced into TCM hospitals from 2012, only reduced conventional drug prices marginally, including the cost of stroke-related drugs, by 2015 [6]. Since Chinese herbal medication was omitted from the zero-markup policy, partly to promote TCM medication use, we suspect that physicians might continue to overprescribe Chinese herbal medicine to pursue their own monetary rewards. We recommend that policymakers regulate the use and pricing of TCM as well as conventional medications to constrain any for-profit overprescribing. In addition, physician training and supervision should promote ethical use of TCM medications, advising patients on costs and benefits of TCM treatments.

A higher proportion of TCM users with ischemic stroke chose primary hospitals to receive medical services, consistent with a study from Taiwan [42]. For those who were admitted to primary hospitals, the total inpatient cost for TCM users was lower than TCM nonusers, though not statistically significant. Patients in the rehabilitation or recovery phase of ischemic stroke were more willing to seek medical treatment in primary hospitals [42].

Average length of hospital stay (ALOS) among TCM nonusers was significantly longer than TCM users in our study. On one hand, severe ischemic stroke patients, measured by longer hospital stays and a higher proportion of admission to tertiary hospitals (characterized by advanced clinical capability), may have had less opportunity to use TCM [43]. On the other hand, there was a higher proportion of UEBMI beneficiaries among TCM nonusers. UEBMI beneficiaries usually enjoyed higher reimbursement rate and more comprehensive insurance coverage, and thus they tended to seek more medical treatment and increase their length of stay [31]. Alternatively, the shorter TCM users' ALOS may reflect the efficacy of TCM treatments. Future studies should investigate the role of ALOS in TCM user and TCM nonuser treatments.

There are a number of limitations to this study. First, the claims database could not directly provide evidence for the efficacy of TCM and clinical outcomes of treating ischemic stroke patients. Second, the severity of disease, an important factor influencing the use of TCM and its cost, was controlled using proxy indicators of the presence of comorbidities. Collecting data from patient clinical records would allow the severity of stroke to be assessed. Third, our study only analyzed the impact of prescription of TCM drugs on inpatient cost, including Chinese herbal medicine, Chinese patent medicine, and Chinese medicine injection. Other conventional TCM services like acupuncture and massage were attributed to nonpharmacy services in our study. Lastly, our study contained data in 2015 only. The post-2016 health care reforms, like the full implementation of the zero-drug markup policy, were likely to impact our results. While our sample is a representative sample of 2015 urban ischemic stroke patients, we are cautious about generalizing our results to other diseases.

## 5. Conclusion

Although TCM medication use lowered the cost of conventional medicine compared with TCM nonusers, the total inpatient cost for TCM users was significantly higher than TCM nonusers. The additional costs of ischemic stroke TCM users were due to the extra cost component of TCM medication imposed on top of conventional medication costs. We found that TCM medication costs were positively associated with conventional medication costs, suggesting that TCM mainly played a complementary, not substitute, role to conventional medicine in ischemic stroke treatment in mainland China.

## Figures and Tables

**Table 1:** Sample characteristics of TCM users and TCM nonusers among stroke patients.

Characteristics		Overall	TCM nonusers	TCM users	*P* value
Number of patients, *n* (%)		47321 (100.0)	3478 (7.4)	43843 (92.6)	
Sex, *n* (%)	Male	26795 (56.6)	2098 (60.3)	24697 (56.3)	<0.001
	Female	20526 (43.4)	1380 (39.7)	19146 (43.7)	
Age (years), median (IQR)		68 (61–77)	68 (60–77)	68 (61–76)	0.565
Age group, *n* (%)	0–29	55 (0.1)	12 (0.3)	43 (0.1)	<0.001
	30–44	921 (1.9)	85 (2.4)	836 (1.9)	
	45–59	9245 (19.5)	697 (20.0)	8548 (19.5)	
	60–69	14974 (31.6)	1061 (30.5)	13913 (31.7)	
	70–79	14528 (30.7)	962 (27.7)	13566 (30.9)	
	≧80	7598 (16.1)	661 (19.0)	6937 (15.8)	
Insurance type, *n* (%)	UEBMI	29950 (63.3)	2456 (70.6)	27494 (62.7)	<0.001
	URBMI	17371 (36.7)	1022 (29.4)	16349 (37.3)	
Hospital level, *n* (%)	Primary	9078 (19.2)	500 (14.4)	8578 (19.6)	<0.001
	Secondary	22957 (48.5)	1596 (45.9)	21361 (48.7)	
	Tertiary	15286 (32.3)	1382 (39.7)	13904 (31.7)	
TCM hospital, *n* (%)	Yes	7000 (14.8)	388 (11.2)	6612 (15.1)	<0.001
	No	40321 (85.2)	3090 (88.8)	37231 (84.9)	
Region, *n* (%)	East	16637 (35.2)	1409 (40.5)	15228 (34.7)	<0.001
	Central	21970 (46.4)	1488 (42.8)	20482 (46.7)	
	West	8714 (18.4)	581 (16.7)	8133 (18.6)	
Comorbidity, *n* (%)	Hypertension	2458 (5.2)	92 (2.6)	2366 (5.4)	<0.001
	Coronary heart disease	1558 (3.3)	44 (1.3)	1514 (3.5)	<0.001
	Diabetes	868 (1.8)	44 (1.3)	824 (1.9)	0.009
	Chronic pulmonary disease	394 (0.8)	13 (0.4)	381 (0.9)	0.002
	Peripheral vascular disease	177 (0.4)	7 (0.2)	170 (0.4)	0.083
	Other neurological diseases	168 (0.4)	5 (0.1)	163 (0.4)	0.03
	Rheumatoid arthritis	91 (0.2)	7 (0.2)	84 (0.2)	0.9
	Peptic ulcer disease	87 (0.2)	0 (0.0)	87 (0.2)	0.009
Average length of stay (ALOS)		15.3	17.7	15.1	<0.001

*P* values are based on the chi-square test and Mann–Whitney test; TCM: traditional Chinese medicine, UEBMI: Urban Employee Basic Medical Insurance scheme, URBMI: Urban Resident Basic Medical Insurance scheme, and IQR: interquartile range.

**Table 2:** Inpatient medical cost TCM users and TCM nonusers.

Characteristics		TCM nonusers		TCM users		*P* value
		Median	IQR	Median	IQR	
Sex	Male	6766	(3599–12565)	8032	(4602–14418)	<0.001
	Female	6046	(3371–11126)	7090	(4117–12300)	<0.001
Age group	0–29	7968	(6630–12072)	10348	(4775–19859)	0.299
	30–44	5746	(3257–11238)	7988	(4195–14657)	0.013
	45–59	6468	(3571–12120)	7395	(4210–12867)	<0.001
	60–69	6061	(3336–10996)	7092	(4134–12338)	<0.001
	70–79	6207	(3323–11153)	7751	(4522–13547)	<0.001
	≧80	7583	(4031–15621)	8667	(4813–16331)	0.001
Insurance type	UEBMI	7361	(4039–13210)	9091	(5432–15839)	<0.001
	URBMI	4538	(2541–8500)	5524	(3213–9582)	<0.001
Hospital level	Primary	3570	(1776–9283)	3516	(2115–6070)	0.588
	Secondary	4883	(3040–8539)	6982	(4488–11116)	<0.001
	Tertiary	9595	(5971–15471)	12685	(7977–20786)	<0.001
Admission to TCM hospital	Yes	4663	(3117–8237)	9424	(5909–16751)	<0.001
	No	6786	(3574–12376)	7275	(4157–12840)	<0.001
Region	East	5086	(2050–10609)	6948	(4025–12386)	<0.001
	Central	4928	(3150–8784)	6386	(3870–10606)	<0.001
	West	9092	(5143–15545)	10351	(5882–17599)	<0.001
Comorbidity	Hypertension	7619	(4982–18733)	12178	(7197–21065)	0.001
	Coronary heart disease	7286	(3791–13955)	12497	(7199–22242)	<0.001
	Diabetes	7696	(4494–22358)	14412	(8725–25169)	0.022
	Chronic pulmonary disease	12431	(6664–23773)	17396	(9646–35066)	0.279
	Peripheral vascular disease	12708	(4163–35509)	14008	(9152–25808)	0.572
	Other neurological diseases	4163	(2627–6994)	12976	(8433–19486)	0.002
	Rheumatoid arthritis	6256	(2605–7141)	7388	(4004–13998)	0.14
	Peptic ulcer disease	-	-	16816	(10206–25507)	-

*P* values are based on the Mann–Whitney test; TCM: traditional Chinese medicine; UEBMI: Urban Employee Basic Medical Insurance scheme; URBMI: Urban Resident Basic Medical Insurance scheme; IQR: Interquartile range.

**Table 3:** Multiple regression analysis for total inpatient costs.

Parameters		Coef.	*P* > *z*	95% Wald confidence interval	
				Lower	Upper
Use of TCM	TCM users	0.325	<0.001	0.304	0.347
Length of stay		0.756	<0.001	0.748	0.764
Age		0.002	<0.001	0.002	0.003
Sex	Male	0.026	<0.001	0.015	0.037
Insurance type	UEBMI	0.109	<0.001	0.097	0.121
Hospital type	Tertiary hospital	1.001	<0.001	0.984	1.018
	Secondary hospital	0.535	<0.001	0.520	0.550
Admission to TCM hospitals		−0.006	0.458	−0.022	0.010
Region	East	0.217	<0.001	0.201	0.234
	Central	−0.108	<0.001	−0.124	−0.093
Hypertension		0.054	0.001	0.023	0.085
Coronary heart disease		0.054	0.005	0.016	0.092
Diabetes		0.114	<0.001	0.068	0.159
Chronic pulmonary disease		0.364	<0.001	0.301	0.427
Peripheral vascular disease		0.080	0.091	−0.013	0.172
Other neurological diseases		−0.014	0.781	−0.110	0.083
Rheumatoid arthritis		0.034	0.600	−0.092	0.160
Peptic ulcer disease		0.112	0.096	−0.020	0.244
_Cons		5.959	<0.001	5.912	6.006

*R*-square = 0.5780 and adjusted R-square = 0.5779 in a multiple linear regression model that was adjusted for length of stay, age, sex, insurance type, hospital type, region, hypertension, coronary heart disease, diabetes, chronic pulmonary disease, peripheral vascular disease, other neurological diseases, rheumatoid arthritis, and peptic ulcer disease. The baseline represents the inpatient cost for a female who did not use any TCM with Urban Resident Basic Medical Insurance admitted to a primary hospital and non-TCM hospital in the western region without the above-observed comorbidities. TCM: traditional Chinese medicine; UEBMI: Urban Employee Basic Medical Insurance scheme; URBMI: Urban Resident Basic Medical Insurance scheme.

**Table 4:** Composition of medication and medical cost TCM users and TCM nonusers.

Variables		TCM nonusers	TCM users	*P* value
Total medical cost	Median	6455	7579	<0.001
	IQR	(3494–11932)	(4364–13404)	
Total medication cost	Median	2716	4175	<0.001
	IQR	(1155–5463)	(2261–7783)	
	Percentage	45.1	54.6	
Conventional medication cost	Median	2716	2087	<0.001
	IQR	(1155–5463)	(865–4602)	
	Percentage	45.1	32.7	
TCM cost	Median	—	1803	<0.001
	IQR	—	(810–3316)	
	Percentage	—	21.9	
Nonpharmacy cost	Median	3347	3173	0.290
	IQR	(1653–6235)	(1720–5703)	
	Percentage	54.9	45.4	

*P* values are based on the Mann–Whitney test; TCM: traditional Chinese medicine; IQR: interquartile range.

**Table 5:** Multiple regression analysis for TCM cost.

Parameters		Coef.^a^	*P* > *z*	95% Wald confidence interval	
				Lower	Upper
Conventional medication cost		0.144	<0.001	0.132	0.156
Length of stay		0.636	<0.001	0.616	0.657
Age		−0.002	<0.001	−0.003	−0.001
Sex	Male	−0.004	0.769	−0.027	0.020
Insurance type	UEBMI	0.109	<0.001	0.083	0.134
Hospital type	Tertiary hospital	−0.012	0.542	−0.052	0.027
	Secondary hospital	−0.113	<0.001	−0.147	−0.080
Admission to TCM hospitals		0.225	<0.001	0.192	0.258
Region	East	−0.006	0.712	−0.040	0.028
	Central	−0.129	<0.001	−0.161	−0.097
Hypertension		−0.045	0.162	−0.109	0.018
Coronary heart disease		0.261	<0.001	0.183	0.338
Diabetes		0.068	0.159	−0.027	0.162
Chronic pulmonary disease		−0.120	0.068	−0.249	0.009
Peripheral vascular disease		0.111	0.251	−0.078	0.299
Other neurological diseases		−0.189	0.059	−0.385	0.007
Rheumatoid arthritis		−0.134	0.319	−0.397	0.129
Peptic ulcer disease		−0.474	<0.001	−0.738	−0.209
_Cons		4.771	<0.001	4.670	4.872

^a^ *R*-square = 0.1893 and adjusted *R*-square = 0.1889 in a multiple linear regression model that was adjusted for length of stay, age, sex, insurance type, hospital type, region, hypertension, coronary heart disease, diabetes, chronic pulmonary disease, peripheral vascular disease, other neurological diseases, rheumatoid arthritis, and peptic ulcer disease. The baseline represents the TCM cost for a female with Urban Resident Basic Medical Insurance admitted to a primary hospital and non-TCM hospital in the western region without the above-observed comorbidities. TCM: traditional Chinese medicine; UEBMI: Urban Employee Basic Medical Insurance scheme; URBMI: Urban Resident Basic Medical Insurance scheme.

## Data Availability

The data that support the findings of this study are available from China Health Insurance Research Association but restrictions apply to the availability of these data, which were used under license for the current study and so are not publicly available. Data are however available from the authors upon reasonable request and with permission of the China Health Insurance Research Association.

## Abbreviations

TCM: Traditional Chinese medicine
LOS: Length of stay
UEBMI: Urban Employee Basic Medical Insurance
URBMI: Urban Resident Basic Medical Insurance
IQR: Interquartile range.
